# A meta-analysis and of clinical values of 11 blood biomarkers, such as AFP, DCP, and GP73 for diagnosis of hepatocellular carcinoma

This article has been retracted.

**DOI:** 10.1080/07853890.2022.2153163

**Published:** 2022-12-08

**Authors:** Bing-yao Pang, Yan Leng, Xiaoli Wang, Yi-qiang Wang, Li-hong Jiang

**Affiliations:** a Changchun University of Traditional Chinese Medicine, Changchun, Jilin, China; b Department of Hepatology, The Affiliated Hospital of Changchun University of Traditional Chinese Medicine, Changchun, Jilin, China; c Department of Cardiology, The Affiliated Hospital of Changchun University of Traditional Chinese Medicine, Changchun, Jilin, China

**Keywords:** Biomarkers, HCC, the diagnostic value, meta-analysis

## Abstract

**Background:**

Hepatocellular carcinoma lacks ideal diagnostic biomarkers. There is a lack of scientific evaluation of relevant promising biomarkers as well. Therefore this study reanalyzes the related studies of 11 blood biomarkers of HCC, and compares the diagnostic value of these biomarkers for HCC systematically.

**Methods:**

The relevant literatures on the diagnostic value in HCC of 11 blood indexes in recent 5 years were searched in PubMed, Embase, and Cochrane libraries. Data were extracted and analyzed.

**Results:**

Finally, 83 literature studies were brought into meta-analysis. The pooled sensitivity and specificity of AFP were 0.61 and 0.87, respectively. The AUC of AFP were 0.78. The AUC and sum of sensitivity and specificity of the combination of AFP and other biomarkers were all significantly higher than that of AFP, including AFP + AFP-L3 + DCP, AFP + DCP, AFP/DCP, AFP + GPC3. Among other biomarkers, the AUC and sum of sensitivity and specificity of biomarkers including DCP, GPC3, GP73, Hsp90alpha, midkine, and OPN were significantly higher than that of AFP. In this study, GP73 had the highest sum of sensitivity and specificity (1.78) and AUC (0.95).

**Conclusions:**

The pooled sensitivity and specificity of AFP were 0.61 and 0.87, respectively. The AUC of AFP were 0.78. The combination of AFP and other biomarkers improved the diagnostic efficiency. The diagnostic value of biomarkers including DCP, GPC3, GP73, Hsp90alpha, midkine, and OPN was higher than that of AFP. GP73 had the best diagnostic value for HCC with the highest sum of sensitivity and specificity (1.78) and AUC (0.95).

**KEY MESSAGES**
- The pooled sensitivity and specificity of AFP were 0.61 and 0.87, respectively. The AUC of AFP were 0.78. The combination of AFP and other biomarkers improved the diagnostic efficiency of HCC.
- The diagnostic value of biomarkers including DCP, GPC3, GP73, Hsp90alpha, midkine, and OPN was higher than that of AFP.
- GP73 had the best diagnostic value for HCC.

## 1. Introduction

Hepatocellular carcinoma(HCC) has become an important public health problem worldwide because of its high mortality [1]. In Asia, HCC secondary to hepatitis B virus is more common. HCC secondary to alcoholic liver disease is also increasing in western developed countries. Due to the symptoms of HCC are not obvious in the early stage, many patients are in the advanced stage when diagnosed, missing the best opportunity for treatment. The early diagnosis of HCC can not only improve the survival time and quality of life of patients but also save the cost of treatment. Therefore, the early diagnosis is the breakthrough focus of HCC treatment.

Alpha fetoprotein (AFP) is the most commonly used biomarker for the diagnosis of HCC, but the diagnostic value of AFP is gradually being doubted because of its low sensitivity, especially for early HCC [2]. Many studies were devoted to finding biomarkers with better diagnostic value in HCC [3].

Recently, many new biomarkers attracted public attention, such as AFP-L3, DCP, DKKI, GP73, and so on. Alpha-fetoprotein-L3(AFP-L3), as a heterogeneous body of AFP, mainly comes from HCC cells. Des-γ-carboxyprothrombin (DCP), also known as protein induced by vitamin K absence or antagonist II (PIVKAII), can appear in the serum of patients with vitamin K absence or HCC [4]. Dickkopf-1 (DKK1) is a secretory glycoprotein that inhibits Wnt signalling pathway by binding to Wnt receptor LRP5/6 [5]. Wnt signalling pathway is an important mechanism for the occurrence and development of HCC and other tumours. Golgi protein 73 (GP73), a type II transmembrane glycoprotein resident in golgi apparatus, is expressed in a small amount in normal liver while it can be specifically expressed, especially around connective tissue and cirrhotic nodules, when liver diseases, such as HCC occur [6]. Glypican-3 (GPC3) is a heparan sulphate glycoprotein on the surface of cell membrane, which is a specific antigen related to HCC [7]. Osteopontin (OPN) is a kind of protein, widely distributed in a variety of tissues and cells. It can participate in tissue repair, self-metabolism, and other functions. The expression level of OPN is closely related to the clinicopathological features of HCC, such as envelope infiltration, vascular invasion, lymph node metastasis, and clinical stage [8,9]. A-L-fucosidase (AFU) is an acidic hydrolase, which is mainly involved in the catabolism of macromolecular substances containing fucosyl, such as glycolipids, glycoproteins, mucopolysaccharides. Junna reported the over expression of AFU in the serum of patients with primary HCC, suggesting that AFU might be a potential marker for the early diagnosis of HCC [10]. Carbohydrate antigen199 (CA199), glycolipid on cell membrane is a kind of glycoprotein antigen that can recognize tumour specific macromolecules [11,12]. Heat shock protein 90alpha (Hsp90alpha) is a multifunctional molecular chaperone, which is widely involved in physiological activities, such as cell signal transduction, hormone response, and transcriptional regulation, maintaining the normal physiological function of cells [13]. Hsp90alpha keeps silent in normal cells while active in tumour cells. Midkine (MDK) is a secretory cytokine, which can participate in the occurrence and development of malignant tumours by promoting division, promoting angiogenesis, and antiapoptosis [14,15]. In recent years, there were more and more studies on the diagnostic value of the above biomarkers for HCC, so which biomarker had a better diagnostic value?

In this study, the meta-analysis was used to reanalyze the related studies of 11 biomarkers, so as to analyze and compare the diagnostic value of biomarkers for HCC more systematically and scientifically.

## 2. Materials and methods

### 2.1. Literature search

This meta-analysis followed Preferred Reporting Items for Systematic Reviews and Meta-analysis (PRISMA) Guidelines. The relevant literatures on the diagnostic value of 11 blood indexes, such as AFP, AFP-L3, and DCP in HCC in recent 5 years were comprehensively and systematically searched in PubMed, Embase, and Cochrane libraries. The keywords used for retrieval included three parts: (1) (AFP OR alpha-fetoprotein) OR (AFP-L3 OR alpha-fetoprotein-L3 OR lens culinaris-agglutinin-reactive fraction of AFP) OR (PIVKA-II OR DCP OR des-γ-carboxyprothrombin) OR (dickkopf-1 OR DKK1) OR (GP73 OR golgi protein 73) OR (glypican-3 OR GPC3) OR (osteopontin OR OPN) OR (α-L-fucosidase OR AFU) OR (carbohydrate antigen199 OR CA199) OR (heat shock protein 90alpha OR Hsp90alpha) OR (midkine OR MDK) (2) HCC OR hepatocellular carcinoma OR liver cancer OR hepatocellular OR hepatoma (3) sensitivity OR specificity. The above three parts were connected by ‘and’. The retrieved literature was published from January 2017 to January 2022.

### 2.2. Inclusion and exclusion criteria

The inclusion criteria of literature were as follows:

1. The diagnostic value of at least one of the 11 biomarkers was described to ensure that we could extract and calculate key indicators directly or indirectly, including sensitivity, specificity, true positive (TP), false positive (FP), false negative (FN) and true negative (TN);
2. The diagnosis of HCC was based on recognized guidelines, such as histopathology or other appropriate diagnostic criteria;
3. The specimen type was serum;
4. The control group was consisted of patients with chronic liver disease, such as liver cirrhosis or hepatitis, or patients with benign liver disease like liver cyst or healthy people.

The exclusion criteria were defined as follows:

1. The article provided incomplete diagnostic information;
2. Meta analysis, systematic review, case review, case report, letter;
3. The control group involved other malignant tumours, especially gastrointestinal tumours;
4. The article from non-human research;
5. The article with <20 research samples;

### 2.3. Data extraction

Two authors screened each record retrieved and extracted data independently. Any differences were resolved through discussion until a consensus was reached or a third author was consulted. Following information was extracted from qualified Literature: author, year of publication, patient country, comprehensive sensitivity and specificity of biomarkers, TP, FP, FN, and TN, type, and number of cases. Finally, the pooled sensitivity and specificity, diagnostic odds ratio, area under the curve, positive likelihood ratio, and negative likelihood ratio were evaluated.

### 2.4. Statistical analysis

The stata software (midas) was used for meta-analysis. Meta-disc software was used to calculate Spearman’s correlation coefficient values to evaluate the threshold effect. *p* < 0.05 was considered as a significant manifestation of threshold effect. At the same time, the Cochran *Q* test and I-squared test were performed to estimate the existence and severity of heterogeneity. *p* < 0.1, and *I*^2^ > 50% were considered significant manifestations of heterogeneity. The Deeks’ funnel plot was used for publication bias analysis. *p* < 0.05 was considered to have potential publication bias.

## 3. Results

The flow chart of the inclusion and exclusion of studies in the review is shown in Figure 1. As shown in the figure, a total of 1751 documents were retrieved from three databases, of which 620 duplicates were eliminated and 1131 were left. Among the leaving documents, there were 784 unrelated to the subject, 192 reviews or meta-analysis, seven non-human related studies, 20 non serum samples, 23 with incomplete date, six with other malignancies in the control group, 10 without recognized diagnostic guidelines for HCC, and six studies with <20 samples. Finally, 83 studies were included in the meta-analysis.

**Figure 1.** Flow chart of research.

### 3.1. AFP and AFP combined with other biomarkers

Among the 83 literature studies, 43 were related to the diagnostic value of AFP, six were related to AFP + AFP-L3, six were related to AFP + AFP-L3 + DCP, 10 were related to AFP + DCP, six were related to AFP/DCP, and eight were related to AFP + GPC3. In the above multi-biomarker combination types, ‘A + B’ represents series diagnosis, which can be diagnosed as positive if they are all positive, while ‘A/B’ is parallel diagnosis, and one positive item can be diagnosed as positive. The study ID, region, and other research characteristics were summarized in Table 1.

**Table 1.** Main characteristics of the included literature related to AFP and AFP combined with other biomarkers in this study.

Markers	Study id [Ref]	Region	Case/control	Sample size (case/control)	TP	FP	FN	TN	Se (%)	Sp (%)
AFP	Mashaly, A. H. 2018 [14]	Egypt	HCC/CLD	44/31	23	1	21	30	52.27	96.77
	Qian, Y. 2020 [16]	China	HCC/CLD	118/75	68	27	50	48	57.63	64.00
	Lee, J. 2021 [17]	Korea	HCC/CLD	184/134	83	11	101	123	45.00	91.80
	Sultanik, P. 2017 [18]	France	HCC/CLD	46/116	29	21	17	95	63.00	82.00
	Kim, M. N. 2019 [19]	Korea	HCC/CLD	64/328	42	22	22	306	65.60	93.30
	Park, S. J. 2017 [20]	Korea	HCC/CLD	79/77	49	6	30	71	62.03	92.21
	Xu, F. 2021 [21]	China	HCC/CLD	308/60	212	10	96	50	68.80	83.30
	Loglio, A. 2020 [22]	Italy	HCC/CLD	64/148	36	9	28	139	56.00	94.00
	Ye, F. 2021 [23]	China	HCC/CLD	133/101	80	9	53	92	60.15	91.09
	Wang, F. 2021 [24]	China	HCC/CLD	186/235	118	58	68	177	63.40	75.30
	Omran, M. M. 2021 [25]	Egypt	HCC/CLD	155/60	42	0	113	60	27.00	100.00
	Malov, S. I. 2021 [26]	Russia	HCC/CLD	55/55	25	3	30	52	45.50	94.50
	Lambrecht, J. 2021 [27]	Germany	HCC/CLD	122/145	97	31	25	114	79.17	78.87
	Zhou, P. C. 2020 [28]	China	HCC/CLD	20/20	6	0	14	20	30.00	100.00
	Zhang, X. 2020 [29]	China	HCC/CLD	288/286	210	53	78	233	72.90	81.50
	Hendy, O. M. 2020 [30]	Egypt	HCC/CLD	40/30	25	2	15	28	62.50	93.33
	Mao, L. 2017 [31]	China	HCC/CLD	82/29	37	10	45	19	45.12	65.52
	Jasirwan, C. O. 2020 [32]	Indonesia	HCC/CLD	132/198	109	57	23	141	82.60	71.20
	Lee, H. A. 2021 [33]	Korea	HCC/CLD	160/462	126	181	34	281	78.80	61.00
	Yang, M. Y. 2021 [34]	China	HCC/CLD	314/300	194	114	120	186	61.80	62.00
	Schotten, C. 2021 [35]	Germany	HCC/CLD	196/377	119	15	77	362	60.70	96.00
	Liu, D. 2021 [36]	China	HCC/CLD	123/143	65	9	58	134	52.80	93.70
	Omran, M. M. 2020 [37]	Egypt	HCC/CLD	104/92	30	0	74	92	29.00	100.00
	Li, B. 2020 [38]	China	HCC/CLD	104/95	60	13	44	82	57.70	86.30
	Yang, T. 2019 [39]	China	HCC/CLD	289/211	193	44	96	167	66.80	79.20
	Wang, Q. 2019 [40]	China	HCC/CLD	176/359	114	82	62	277	64.80	77.20
	Shimagaki, T. 2019 [41]	Japan	HCC/CLD	185/108	93	16	92	92	50.30	85.20
	Hu, J. 2018 [42]	China	HCC/CLD	369/176	213	26	156	150	57.70	85.20
	Guo, W. 2018 [43]	China	HCC/CLD	200/101	114	20	86	81	57.00	80.00
	Chuaypen, N. 2018 [44]	Thailand	HCC/CLD	150/150	97	4	53	146	64.70	97.30
	Tian, M. M. 2017 [45]	China	HCC/CLD	120/146	66	56	54	90	55.00	61.60
	Shaker, M. K. 2017 [46]	Egypt	HCC/CLD	50/25	35	1	15	24	70.00	96.00
	Ismail, M. M. 2017 [47]	Saudi Arabia	HCC/CLD	66/99	45	12	21	87	68.20	87.90
	Hu, N. 2017 [48]	China	HCC/CLD	80/80	47	20	33	60	58.75	75.00
	Fu, Y. 2017 [49]	China	HCC/CLD	531/171	408	29	123	142	76.82	83.01
	Liu, H. H. 2020 [50]	China	HCC/CLD	105/54	38	5	67	49	36.19	90.74
	Tang, X. Q. 2017 [51]	China	HCC/CLD	176/190	130	32	46	158	73.90	82.90
	Ali, O. M. 2020 [52]	Egypt	HCC/CLD	30/30	22	4	8	26	72.20	86.20
	Sai, W. L. 2021 [53]	China	HCC/CLD	126/96	93	21	33	75	73.81	78.13
	Alzamzamy, A. 2021 [54]	Egypt	HCC/CLD	40/60	26	10	14	50	65.00	83.30
	Ricco G. 2018 [55]	Italy	HCC/CLD	258/130	135	32	123	98	52.50	75.20
	Caviglia GP. 2021 [56]	Italy	HCC/CLD	72/119	55	37	17	82	76.40	68.90
	Caviglia GP. 2020 [57]	Italy	HCC/CLD	149/200	107	68	42	132	72.00	66.00
AFP + AFP-L3	Song, T. 2020 [58]	China	HCC/CLD	100/67	54	7	46	60	53.50	89.60
	Pan, Y. 2019 [59]	China	HCC/CLD, HC	125/280	72	23	53	257	57.60	91.80
	Hu, R. Z. 2019 [60]	China	HCC/CLD	56/91	36	8	20	83	64.28	90.90
	Park, S. J. 2017 [20]	Korea	HCC/CLD	79/77	35	2	44	75	44.30	97.40
	Choi, J. 2019 [61]	Korea	HCC/CLD	42/168	33	22	9	146	79.00	87.00
	Chen, H. 2018 [62]	China	HCC/CLD	202/441	83	44	119	397	40.90	90.00
AFP + AFP-L3 + DCP	Song, T. 2020 [58]	China	HCC/CLD	100/67	67	11	33	56	66.70	83.10
	Pan, Y. 2019 [59]	China	HCC/CLD, HC	125/280	65	18	60	262	52.00	93.60
	Hu, R. Z. 2019 [60]	China	HCC/CLD	56/91	31	2	25	89	55.35	98.48
	Park, S. J. 2017 [20]	Korea	HCC/CLD	79/77	30	0	49	77	37.97	100.00
	Choi, J. 2019 [61]	Korea	HCC/CLD	42/168	35	42	7	126	83.00	75.00
	Chen, H. 2018 [62]	China	HCC/CLD, HC	202/644	149	64	53	580	73.70	90.00
AFP + DCP	Park, S. J. 2017 [20]	Korea	HCC/CLD	79/77	40	0	39	77	51.00	100.00
	Xu, F. 2021 [21]	China	HCC/CLD, BLD	308/120	293	20	15	100	95.10	83.30
	Yang, T. 2019 [39]	China	HCC/CLD	289/211	254	40	35	171	87.80	81.00
	Wang, Q. 2019 [40]	China	HCC/CLD	176/359	129	22	47	337	73.30	93.90
	Tang, X. Q. 2017 [51]	China	HCC/CLD	176/190	154	25	22	165	87.50	87.00
	Pan, Y. 2019 [59]	China	HCC/CLD, HC	125/280	78	21	47	259	62.00	92.50
	Wu, M. 2020 [63]	China	HCC/CLD, HC	198/176	160	52	38	124	80.80	70.60
	Maeda, T. 2019 [64]	Japan	HCC/CLD, HC	304/152	224	13	80	139	73.70	91.70
	Wu, J. 2018 [65]	China	HCC/CLD, HC	143/131	126	44	17	87	88.10	66.41
	Ricco G. 2018 [55]	Italy	HCC/CLD	258/130	225	62	33	68	87.40	52.20
AFP/DCP	Park, S. J. 2017 [20]	Korea	HCC/CLD	79/77	65	29	14	48	82.28	62.34
	Lee, Q. 2021 [66]	China	HCC/CLD	158/62	114	2	44	60	72.20	96.80
	Loglio, A. 2020 [22]	Italy	HCC/CLD	64/148	51	21	13	127	80.00	86.00
	Sultanik, P. 2017 [18]	France	HCC/CLD	46/116	40	28	6	88	87.00	76.00
	Wu, J. 2018 [65]	China	HCC/CLD, HC	143/131	76	9	67	122	53.02	93.13
	Pan, Y. 2019 [59]	China	HCC/CLD, HC	125/280	114	53	11	227	91.20	81.10
AFP + GPC3	Wu, M. 2020 [63]	China	HCC/CLD, HC	198/176	172	50	26	126	86.90	71.70
	Zhu, X. 2019 [67]	China	HCC/CLD	47/89	40	16	7	73	85.01	81.62
	Taketomi, A. 2020 [68]	Egypt	HCC/CLD, HC	25/125	23	0	2	125	92.00	100.00
	Tang, X. Y. 2020 [69]	China	HCC/HC, BLD	166/144	146	32	20	112	87.82	77.86
	Shimizu, Y. 2020 [70]	Japan	HCC/CLD	105/95	72	10	33	85	68.30	89.40
	Liu, S. 2020 [71]	China	HCC/HC	210/127	185	22	25	105	88.10	82.68
	Sun, B. 2017 [7]	China	HCC/CLD, HC	76/100	65	4	11	96	85.50	96.00
	Ali, O. M. 2020 [52]	Egypt	HCC/CLD	30/30	27	4	3	26	91.00	86.00

CLD: chronic liver disease; BLD: benign liver disease; HC: healthy control; CH: cirrhosis; TP: true positive; FP: false positive; FN: false negative; TN: true negative; Se: sensitivity; Sp: specificity; Ref: reference.

We combined the data from individual diagnostic tests for AFP and data from the study on combined analysis of AFP and other biomarkers. The sensitivity and specificity after combination are shown in Figure 2, and the SROC curve is shown in Figure 3. Forty-three literatures related to AFP in recent 5 years were included in the study. The pooled sensitivity and specificity of AFP were 0.61 and 0.87, respectively. The AUC of AFP were 0.78. To better compare the diagnostic value, we compared the sum of sensitivity and specificity.

**Figure 2.** The sensitivity and specificity of AFP and its combined with other biomarkers (A, AFP; B, AFP + AFP-L3; C, AFP + AFP-L3 + DCP; D, AFP + DCP; E, AFP/DCP; F, AFP + GPC3).

**Figure 3.** The SROC curve of AFP and its combined with other biomarkers (A, AFP; B, AFP + AFP-L3; C, AFP + AFP-L3 + DCP; D, AFP + DCP; E, AFP/DCP; F, AFP + GP73).

Among studies on combined analysis of AFP and other biomarkers, the sum of sensitivity and specificity of AFP + AFP-L3 + DCP was significantly higher than that of AFP, as were AFP + DCP, AFP/DCP, and AFP + GPC3. The AUC of AFP + AFP-L3, AFP + AFP-L3 + DCP, AFP + DCP, AFP/DCP, and AFP + GPC3 were higher than that of AFP. The combination of AFP and other biomarkers improved the diagnostic efficiency. AFP + GPC3 had the highest sum of sensitivity and specificity (1.75) and AUC (0.91). The pooled sensitivity, specificity, diagnostic odds ratio, area under the curve, positive likelihood ratio, and negative likelihood ratio are shown in Table 2.

**Table 2.** The pooled sensitivity, specificity, diagnostic odds ratio, area under the curve, positive likelihood ratio, and negative likelihood ratio of AFP and AFP combined with other biomarkers.

Markers	Sensitivity (95% CI)	Specificity (95% CI)	PLR (95% CI)	NLR (95% CI)	DOR (95% CI)	AUC
AFP	0.61 [0.57, 0.65]	0.87 [0.83, 0.90]	4.50 [3.60, 5.80]	0.45 [0.41, 0.49]	10.00 [8.00, 13.00]	0.78
AFP + AFP-L3	0.56 [0.45, 0.66]	0.90 [0.88, 0.92]	5.80 [4.70, 7.31]	0.49 [0.39, 0.61]	12.00 [8.00, 18.00]	0.90
AFP + AFP-L3 + DCP	0.62 [0.49, 0.74]	0.93 [0.84, 0.97]	9.00 [4.50, 17.90]	0.40 [0.30, 0.54]	22.00 [13.00, 38.00]	0.85
AFP + DCP	0.81 [0.73, 0.88]	0.86 [0.75, 0.93]	6.00 [3.40, 10.60]	0.21 [0.15, 0.30]	28.00 [17.00, 47.00]	0.90
AFP/DCP	0.80 [0.68, 0.88]	0.85 [0.74, 0.92]	5.30 [3.20, 8.90]	0.24 [0.16, 0.36]	22.00 [13.00, 38.00]	0.89
AFP + GPC3	0.86 [0.80, 0.90]	0.89 [0.79, 0.95]	8.10 [3.80, 17.20]	0.16 [0.12, 0.22]	50.00 [20.00, 127.00]	0.91

PLR: positive likelihood ratio; NLR: negative likelihood ratio; DOR: diagnostic odds ratio; CI: confidence interval; AUC: area under the curve.

We used meta-disc software to calculate Spearman’s correlation coefficient values to evaluate the threshold effect. Spearman’s relevance coefficient value was 0.407 (*p* = 0.154) in AFP, 0.371 (*p* = 0.468) in AFP + AFP-L3, 0.886 (*p* = 0.089) in AFP + AFP-L3 + DCP, 0.717 (*p* = 0.224) in AFP + DCP, 0.714 (*p* = 0.111) in AFP/DCP, −0.190 (*p* = 0.651) in AFP + GPC3. There was no threshold effect in the analysis of each group.

Cochran *Q* test and *I*-squared test were performed to estimate the existence and severity of heterogeneity. *p* < 0.1, and *I*^2^ > 50% were considered significant manifestations of heterogeneity. It was found that AFP + AFP-L3 + DCP, AFP, AFP + AFP-L3, AFP + DCP, AFP/DCP, and AFP + GPC3 was heterogeneous.

Meta-regression analysis was performed to analyze the sources of heterogeneity. Potential sources of heterogeneity included research time, publication time, race, average age of HCC group, male proportion of HCC group, proportion of early HCC, male proportion of control group, and average age of control group. The source of heterogeneity of AFP also included cut-off values. The inclusion studies of AFP + AFP-L3, and AFP + AFP-L3 + DCP were all from the same race. The results were shown in Figure 4.

**Figure 4.** The univariable meta-regression and subgroup analysis of AFP and its combined with other biomarkers (A, AFP; B, AFP + AFP-L3; C, AFP + AFP-L3 + DCP; D, AFP + DCP; E, AFP/DCP; F, AFP + GPC3) (year1, research time; year2, publication time; age1, average age of HCC group; male1, male proportion of HCC group; *n*, proportion of early HCC; male2, male proportion of control group; age2, average age of control group).

As shown in Figure 4, the meta-regression results of AFP + AFP-L3 showed that the heterogeneity of AFP + AFP-L3 sensitivity may be derived from the male proportion of HCC group, the heterogeneity of AFP + AFP-L3 + DCP specificity may be derived from the male proportion of HCC group and control group, the heterogeneity of AFP/DCP sensitivity may be derived from the early HCC proportion of HCC group, and the heterogeneity of specificity may be derived from the male proportion of HCC group. The source of heterogeneity in other groups was not found.

The sensitivity analysis results were shown in Figure 5. It could be seen from the figure that the meta-analysis results of all markers were relatively stable.

**Figure 5.** The sensitivity analysis of AFP and its combined with other biomarkers (A, AFP; B, AFP + AFP-L3; C, AFP + AFP-L3 + DCP; D, AFP + DCP; E, AFP/DCP; F, AFP + GPC3).

We used stata software to analyze the potential publication bias of each group. There was no potential publication bias in each group.

### 3.2. Other biomarkers

Among the 83 literature studies, four were related to AFU, seven were related to AFP-L3, five were related to CA199, 19 were related to DCP, six were related to DKK1, nine were related to GP73, eight were related to GPC3, four were related to Hsp90alpha, five were related to midkine, four were related to OPN, The study ID, region and other research characteristics were summarized in Table 3.

**Table 3.** Main characteristics of the included literature related to other biomarkers in this study.

Markers	Study id [Ref]	Region	Case/control	Sample size (case/control)	TP	FP	FN	TN	Se (%)	Sp (%)
DCP	Lee, H. A. 2021 [33]	Korea	HCC/CLD	160/462	100	20	60	442	62.50	96.00
	Park, S. J. 2017 [20]	Korea	HCC/CLD	79/77	56	23	23	54	70.89	70.13
	Xu, F. 2021 [21]	China	HCC/CLD, BLD	308/120	274	10	34	110	89.00	91.70
	Loglio, A. 2020 [22]	Italy	HCC/CLD	64/148	41	13	23	135	64.00	91.00
	Malov, S. I. 2021 [26]	Russia	HCC/CLD	55/55	30	6	25	49	54.60	88.60
	Yang, T. 2019 [39]	China	HCC/CLD	289/211	229	17	60	194	79.00	91.90
	Wang, Q. 2019 [40]	China	HCC/CLD	176/359	143	23	33	336	81.30	93.60
	Shimagaki, T. 2019 [41]	Japan	HCC/CLD	185/108	122	14	63	94	66.00	87.00
	Lee, J. 2021 [17]	Korea	HCC/CLD	184/134	68	6	116	128	37.00	95.50
	Ji, J. 2021 [72]	China	HCC/CLD	183/601	154	58	29	543	84.08	90.43
	Tang, X. Q. 2017 [51]	China	HCC/CLD	176/190	145	8	31	182	82.40	95.90
	Sultanik, P. 2017 [18]	France	HCC/CLD	46/116	34	9	12	107	74.00	92.00
	Wu, J. 2018 [65]	China	HCC/CLD, HC	143/131	110	18	33	113	76.92	86.26
	Pan, Y. 2019 [59]	China	HCC/CLD, HC	125/280	101	26	24	254	80.80	90.70
	Ao, J. 2021 [73]	Japan	HCC/CLD, HC	275/118	170	4	105	114	61.80	96.90
	Wu, M. 2020 [63]	China	HCC/CLD, HC	198/176	59	5	139	171	29.80	97.20
	Caviglia GP. 2020 [57]	Italy	HCC/HC	149/200	101	32	48	168	68.00	84.00
	Caviglia GP. 2021 [56]	Italy	HCC/CLD	72/119	54	17	18	102	75.00	85.70
	Ricco G. 2018 [55]	Italy	HCC/CLD	258/130	203	49	55	81	78.70	62.50
GPC3	Malov, S. I. 2021 [26]	Russia	HCC/CLD	55/55	33	2	22	53	60.00	96.40
	Jing, J. S. 2017 [74]	China	HCC/CLD	39/31	35	1	4	30	89.70	96.77
	Wang, Y. Y. 2017 [75]	China	HCC/CLD	60/50	39	3	21	47	65.00	94.00
	Wu, M. 2020 [63]	China	HCC/CLD, HC	198/176	116	28	82	148	58.60	84.40
	Liu, S. 2020 [71]	China	HCC/HC	210/134	167	20	43	114	79.52	85.07
	Sun, B. 2017 [7]	China	HCC/CLD, HC	76/100	57	13	19	87	75.00	87.00
	Caviglia GP. 2020 [57]	Italy	HCC/HC	149/200	109	98	40	102	73.00	51.00
	Caviglia GP. 2021 [56]	Italy	HCC/CLD	72/119	45	21	27	98	62.50	82.40
GP73	Wei, H. 2020 [76]	China	HCC/CLD	60/60	48	35	12	25	80.00	41.70
	Malov, S. I. 2021 [26]	Russia	HCC/CLD	55/55	35	11	20	44	63.60	80.00
	Jing, J. S. 2017 [74]	China	HCC/CLD	39/31	36	5	3	26	92.31	83.87
	Ismail, M. M. 2017 [47]	Saudi Arabia	HCC/CLD	66/99	66	0	0	99	100.00	100.00
	Farag, R. M. 2019 [77]	Saudi Arabia	HCC/CLD, HC	145/155	138	8	7	147	95.00	95.00
	Wu, M. 2020 [63]	China	HCC/CLD, HC	198/176	47	1	151	175	23.70	99.40
	Yanming, L. 2019 [78]	China	HCC/CLD, HC	93/628	71	125	22	503	76.34	80.09
	Elzefzafy, W.M. 2021 [79]	Egypt	HCC/CLD, HC	30/60	29	27	1	33	95.00	55.00
DKK1	Piratvisuth, T. 2022 [80]	Thailand	HCC/CLD	308/773	67	77	241	696	21.60	90.00
	Mao, L. 2017 [31]	China	HCC/CLD	82/57	73	32	9	25	89.02	43.86
	ElShayeb, A. F. 2021 [81]	Egypt	HCC/CLD	86/89	77	18	9	71	89.00	80.00
	Eldeeb, M. K. 2020 [82]	Egypt	HCC/CLD	30/30	12	3	18	27	40.00	90.00
	Awad, A. E. 2019 [83]	Egypt	HCC/CLD, HC	55/35	48	6	7	29	87.30	82.90
	Zhu, M. 2020 [8]	China	HCC/CLD	101/221	65	80	36	141	64.36	63.80
AFP-L3	Lee, H. A. 2021 [33]	Korea	HCC/CLD	160/462	114	90	46	372	71.30	81.00
	Song, T. 2020 [58]	China	HCC/CLD	100/67	28	3	72	64	28.30	95.50
	Park, S. J. 2017 [20]	Korea	HCC/CLD	79/77	40	13	39	64	50.63	83.12
	Malov, S. I. 2021 [26]	Russia	HCC/CLD	55/55	16	2	39	53	29.10	96.40
	Pan, Y. 2019 [59]	China	HCC/CLD, HC	125/280	88	24	37	256	70.40	91.40
	Liu, R. 2021 [84]	China	HCC/CLD, HC	89/119	66	12	23	107	74.20	89.90
	Yanming, L. 2019 [78]	China	HCC/CLD, HC	93/628	63	116	30	512	67.74	81.52
AFU	Liu, D. 2021 [36]	China	HCC/CLD	123/143	88	47	35	96	71.50	67.10
	Xing, H. 2019 [85]	China	HCC/CLD	187/214	124	98	63	116	66.31	54.21
	Junna, Z. 2017 [10]	China	HCC/HC	36/36	28	13	8	23	78.00	64.00
	ElShayeb, A. F. 2021 [81]	Egypt	HCC/CLD	86/89	64	45	22	44	74.00	50.00
CA199	Li, H. 2020 [11]	China	HCC/CLD	86/85	71	31	15	54	82.94	63.95
	Han, Y. 2021 [86]	China	HCC/CH, BLD	118/62	58	11	60	51	48.90	81.50
	Piratvisuth, T. 2022 [80]	Thailand	HCC/CLD	308/773	99	77	209	696	32.00	90.00
	Huang, X. 2018 [87]	China	HCC/CH	62/40	42	13	20	27	68.43	68.36
	Zhao, L. 2017 [88]	China	HCC/CH, BLD	149/178	24	16	125	162	16.10	90.80
Hsp90alpha	Han, Y. 2021 [86]	China	HCC/CH, BLD	118/62	113	15	5	47	95.70	75.00
	Fu, Y. 2017 [49]	China	HCC/CLD, HC	531/743	496	72	35	671	93.32	90.27
	Wei, W. 2020 [13]	China	HCC/HC	659/230	442	22	217	208	67.07	90.43
	Tang, Y. 2020 [89]	China	HCC/CH, BLD	409/179	297	12	112	167	72.60	93.30
Midkine	Mashaly, A. H. 2018 [14]	Egypt	HCC/CLD	44/31	36	5	8	26	81.82	83.87
	Omran, M. M. 2020 [37]	Egypt	HCC/CLD	104/92	79	19	25	73	76.00	79.00
	Hodeib, H. 2017 [90]	Egypt	HCC/CLD, HC	35/105	34	4	1	101	98.40	96.20
	ElShayeb, A. F. 2021 [81]	Egypt	HCC/CLD	86/89	86	9	0	80	100.00	90.00
	Malov, S. I. 2021 [26]	Russia	HCC/CLD	55/55	47	20	8	35	85.50	63.60
OPN	Zhu, M. 2020 [8]	China	HCC/CLD	101/221	80	45	21	176	79.21	79.64
	Al-Zoubi, S. 2017 [91]	Syria	HCC/CLD, HC	26/42	18	7	8	35	69.00	84.00
	Malov, S. I. 2021 [26]	Russia	HCC/CLD	55/55	44	13	11	42	80.00	76.60
	Hodeib, H. 2017 [90]	Egypt	HCC/CLD, HC	35/105	34	5	1	100	97.10	95.30

CLD: chronic liver disease; BLD: benign liver disease; HC: healthy control; CH: cirrhosis; TP: true positive; FP: false positive; FN: false negative; TN: true negative; Se: sensitivity; Sp: specificity; Ref: reference.

We combined the data from individual diagnostic tests for 10 biomarkers. The sensitivity and specificity after combination are shown in Figure 6, and the SROC curve is shown in Figure 7. Compared to AFP, the sum of sensitivity and specificity of DCP was significantly higher, as were GPC3, GP73, Hsp90alpha, midkine, and OPN. In addition, Midkine and GP73 had the highest sum of sensitivity and specificity (1.78).

**Figure 6.** The sensitivity and specificity of other biomarkers (A, DCP; B, GPC3; C, GP73; D, DK-K1; E, AFP-L3; F, AFU; G, CA199; H, Hsp90alpha; I, Midkine, J, OPN).

**Figure 7.** The SROC curve of other biomarkers (A, DCP; B, GPC3; C, GP73; D, DK-K1; E, AFP-L3; F, AFU; G, CA199; H, Hsp90alpha; I, Midkine, J, OPN).

Taking AFP as the reference, the results showed that the AUC of DCP, GPC3, GP73, DKK1, AFP-L3, Hsp90alpha, Midkine, and OPN were significantly higher than that of AFP. The AUC of GP73 (0.95) was the highest. The pooled sensitivity, specificity, diagnostic odds ratio, area under the curve, positive likelihood ratio, and negative likelihood ratio are shown in Table 4.

**Table 4.** The pooled sensitivity, specificity, diagnostic odds ratio, area under the curve, positive likelihood ratio, and negative likelihood ratio of other biomarkers.

Markers	Sensitivity (95% CI)	Specificity (95% CI)	PLR (95% CI)	NLR (95% CI)	DOR (95% CI)	AUC
DCP	0.71 [0.64, 0.77]	0.91 [0.87, 0.93]	7.8 [5.70, 10.50]	0.32 [0.26, 0.40]	24.00 [16.00, 36.00]	0.90
GPC3	0.71 [0.63, 0.77]	0.87 [0.77, 0.93]	5.50 [2.90, 10.40]	0.33 [0.26, 0.43]	17.00 [7.00, 37.00]	0.82
GP73	0.88 [0.65, 0.96]	0.90 [0.68, 0.98]	8.90 [2.30, 33.90]	0.14 [0.04, 0.45]	66.00 [9.00, 502.00]	0.95
DKK1	0.70 [0.44, 0.87]	0.77 [0.62, 0.87]	3.10 [2.00, 4.80]	0.39 [0.20, 0.77]	8.00 [3.00, 18.00]	0.81
AFP-L3	0.56 [0.42, 0.70]	0.89 [0.83, 0.94]	5.40 [3.70, 7.70]	0.49 [0.36, 0.66]	11.00 [7.00, 18.00]	0.85
AFU	0.71 [0.66, 0.75]	0.59 [0.51, 0.66]	1.70 [1.40, 2.10]	0.50 [0.40, 0.63]	3.00 [2.00, 5.00]	0.71
CA199	0.50 [0.27, 0.72]	0.83 [0.71, 0.90]	2.90 [2.40, 3.50]	0.61 [0.42, 0.88]	5.00 [3.00, 7.00]	0.78
Hsp90alpha	0.87 [0.69, 0.95]	0.89 [0.84, 0.93]	8.20 [5.60, 11.90]	0.15 [0.06, 0.37]	55.00 [24.00, 126.00]	0.94
Midkine	0.93 [0.76, 0.98]	0.85 [0.73, 0.93]	6.40 [3.10, 13.30]	0.08 [0.02, 0.33]	78.00 [11.00, 582.00]	0.94
OPN	0.85 [0.70, 0.93]	0.85 [0.74, 0.92]	5.60 [2.80, 11.40]	0.18 [0.08, 0.41]	31.00 [7.00, 137.00]	0.91

PLR: positive likelihood ratio; NLR: negative likelihood ratio; DOR: diagnostic odds ratio; CI: confidence interval; AUC: area under the curve.

Spearman’s relevance coefficient value was 0.000 (*p* = 1.000) in AFU, 0.571 (*p* = 0.180) in AFP-L3, 1.220 (*p* = 0.230) in CA199, 0.207 (*p* = 0.395) in DCP, 0.714 (*p* = 0.111) in DKK1, −0.143 (*p* = 0.736) in GP73, −0.286 (*p* = 0.493) in GPC3, 0.800 (*p* = 0.200) in Hsp90alpha, −0.600 (*p* = 0.285) in Midkine, −0.200 (*p* = 0.800) in OPN. There was no threshold effect in the analysis of each group.

Cochran *Q* test and *I*-squared test were performed to estimate the existence and severity of heterogeneity. It was found that AFU, AFP-L3, CA199, DCP, DKK1, GP73, GPC3, Hsp90alpha, Midkine, OPN was heterogeneous.

Meta-regression analysis was performed to analyze the sources of heterogeneity of meta-analysis involving more than five articles. Potential sources of heterogeneity included research time, publication time, race, cut-off values, average age of HCC group, male proportion of HCC group, proportion of early HCC, male proportion of control group, and average age of control group.

As shown in Figure 8, the meta-regression results showed that the heterogeneity of DCP sensitivity may be derived from the male proportion of HCC group and the early HCC proportion of HCC group, the heterogeneity of GPC3 sensitivity may be derived from the male proportion of HCC group, the heterogeneity of GP73 sensitivity may be derived from the male proportion of control group, the heterogeneity of DKK1 sensitivity and specificity may be derived from the male proportion of control group. The source of heterogeneity in other groups was not found.

**Figure 8.** The univariable meta-regression and subgroup analysis of other biomarkers (A, DCP; B, GPC3; C, GP73; D, DKK1; E, AFP-L3) (year1, research time; year2, publication time; age1, average age of HCC group; male1, male proportion of HCC group; *n*, proportion of early HCC; male2, male proportion of control group; age2, average age of control group).

The sensitivity analysis results are shown in Figure 9. It could be seen from the figure that the meta-analysis results of all markers were relatively stable.

**Figure 9.** The sensitivity analysis of other biomarkers (A, DCP; B, GPC3; C, GP73; D, DK-K1; E, AFP-L3; F, AFU; G, CA199; H, Hsp90alpha; I, Midkine, J, OPN).

We used Deeks’ funnel plot to analyze the potential publication bias of each group. Among the analysis of each group, DCP (*p* = 0.05) and GPC3 (*p* = 0.04) have potential publication bias. For the publication bias test results of DCP and GPC3, we further tested the publication bias by using Egger’ funnel plot, Begger’ funnel plot, trim and fill methods. The results are shown in Figure 10.

**Figure 10.** Publication bias analysis of DCP and GPC3 (A, Deeks’ funnel plot; B, Beggs’ funnel plot; C, Egger’ funnel plot; D, filled funnel plot) (Left, DCP; Right, GPC3).

As shown in Figure 10, the Egger test result of DCP is *p* = 0.50, and the Egger test result of GPC3 is *p* = 0.286. We analyzed the analysis results of DCP and GPC3 by the trim and fill method. Seven studies were added to DCP. The combined RR value and 95% effect interval before repair were 5.003 (3.766, 6.240), and the combined RR value and 95% effect interval after repair were 14.885 (3.523, 62.893). Four studies were added to GPC3. The combined RR value and 95% effect interval before repair were 3.606 (2.864, 4.348), and the combined RR value and 95% effect interval after repair were 11.676 (5.443, 25.047). The combined RR value before and after repair showed no significant impact on the study.

## 4. Discussion

The early diagnosis is the key to the treatment of HCC. AFP, as the most commonly used clinical biomarker of HCC, has been questioned for its diagnostic value. However, there is no ideal recognized biomarker of HCC at present [92]. There are more and more studies on new biomarkers with better diagnostic value for HCC, lack of scientific evaluation yet. In view of this, we tried to use meta-analysis to compare 11 biomarkers of HCC which were played more attention by public. According to our investigation, there are few such studies to conduct such a wide range of literature research, screen and evaluate so many biomarkers at the same time.

The pooled sensitivity and specificity of AFP were 0.61 and 0.87, respectively, which were consistent with the results of previous studies. It was found that the combination of AFP and other biomarkers improved the diagnostic efficiency. The sum of sensitivity and specificity of AFP + GP73 was the highest (1.75), and AUC was the highest (0.91) as well.

The sum of sensitivity and specificity of DCP was significantly higher than that of AFP, as were GPC3, GP73, Hsp90alpha, midkine, and OPN. Midkine and GP73 had the highest sum of sensitivity and specificity (1.78), higher than AFP + GP73 in the combination diagnosis of AFP and other biomarkers of HCC. The AUC of DCP, GPC3, GP73, DKK1, AFP-L3, Hsp90alpha, midkine, and OPN were significantly higher than that of AFP and GP73’s (0.95) was the highest. It indicated the above biomarkers had higher diagnostic value for HCC, and expected to become ideal biomarkers for HCC diagnosis, worthy of further research.

GP73 was a type II transmembrane glycoprotein that existed in Golgi apparatus. It was generally believed that GP73 was mainly expressed in bile duct epithelial cells in normal liver, with no or only a small amount of expression in hepatocytes and low serum GP73 level; However, hepatocytes in patients with liver cancer produced a large amount of GP73 and further release it into serum, resulting in a significant increase in serum GP73 level [90].

As a potential biomarker of tumour diagnosis and prognosis, GP73 had become a research hotspot. Previous studies had shown that in the diagnosis of early HCC, the sensitivity of GP73 was 62%, which was much higher than that of AFP (sensitivity was 25%), indicating that GP73 was better than AFP in the diagnosis of early HCC [89]. In a study on the population of China, it was found that the serum GP73 level of liver cancer patients infected with hepatitis B virus was the highest in all detection groups [93]. According to this study, it was shown that in the study, GP73 had the highest AUC (0.95), and sum of sensitivity and specificity (1.78). The data of this study shows that GP73 has the best diagnostic value. but the number of relevant research cases was small, which still needed a lot of clinical data for further support.

The diagnostic value of individual biomarker may not be significantly different from that of multi-biomarker combined assays. Perhaps we can find enough good biomarkers from an individual biomarker instead of focusing on multi-biomarker combined assays.

A large number of case–control studies investigated the diagnostic accuracy of serologic biomarkers; However, only few studies investigated the predictiveness of these biomarkers. Serologic biomarkers that monitor the risk stratification of HCC development in patients are crucial to personalize surveillance strategies and thus to improve early HCC detection by optimizing resource allocation.

Loglio et al. reported that in Caucasian patients with HBV compensatory cirrhosis who received long-term NUC treatment, AFP higher than 7 ng/mL showed excellent specificity (99.6%), indicating the occurrence of HCC within a year [94]. El-Derany MO reported HCC development in NASH was associated with higher serum AFP, IL-13 levels [95]. Choi et al. found that the level of DCP in HCC patients began to increase half a year before diagnosis, and the level of AFP-L3 began to increase one year before diagnosis, but there was no significant change in the control group [61]. Li et al. found that the AFP, AFP-L3, ALT, and AFP-L3/AFP increased significantly in patients with HCC 3 years before the diagnosis of HCC [96]. Shakado suggested that the elevation of AFP and DCP levels at 24 weeks after the completion of IFN and ribavirin therapy were strongly associated with the incidence of HCC irrespective of virological response among Japanese hepatitis C virus-related liver cirrhosis patients [97]. Gatselis et al. reported that the combination of GP73 and the cartilage oligomeric matrix protein (COMP) seems efficient to detect the development of HCC in patients with chronic liver diseases [98].

## 5. Conclusions

The pooled sensitivity and specificity of AFP were 0.61 and 0.87, respectively. The AUC of AFP were 0.78. The combination of AFP and other biomarkers improved the diagnostic efficiency. The diagnostic value of biomarkers including DCP, GPC3, GP73, Hsp90alpha, midkine, OPN was higher than that of AFP. GP73 had the best diagnostic value for HCC with the highest sum of sensitivity and specificity (1.78) and AUC (0.95).

## Data Availability

The authors confirm that the data supporting the findings of this study are available within the article.
